# The Aryl Hydrocarbon Receptor Is Constitutively Active in Advanced Prostate Cancer Cells

**DOI:** 10.1371/journal.pone.0095058

**Published:** 2014-04-22

**Authors:** Oliver Richmond, Maryam Ghotbaddini, Cidney Allen, Alice Walker, Shokouh Zahir, Joann B. Powell

**Affiliations:** 1 Clark Atlanta University Center for Cancer Research and Therapeutic Development (CCRTD), Atlanta, Georgia, United States of America; 2 Clark Atlanta University Department of Biological Sciences, Atlanta, Georgia, United States of America; 3 Shahid Sadoughi University of Medical Sciences and Health Services, Yazd, Iran; Innsbruck Medical University, Austria

## Abstract

**Background:**

Distant prostate cancers are commonly hormone refractory and exhibit increased growth no longer inhibited by androgen deprivation therapy. Understanding all molecular mechanisms contributing to uncontrolled growth is important to obtain effective treatment strategies for hormone refractory prostate cancers (HRPC). The aryl hydrocarbon receptor (AhR) affects a number of biological processes including cell growth and differentiation. Several studies have revealed that exogenous AhR ligands inhibit cellular proliferation but recent evidence suggests AhR may possess intrinsic functions that promote cellular proliferation in the absence of exogenous ligands.

**Methods/Results:**

qRT-PCR and western blot analysis was used to determine AhR mRNA and protein expression in hormone sensitive LNCaP cells as well as hormone refractory DU145, PC3 and PC3M prostate cancer cell lines. LNCaP cells express AhR mRNA and protein at a much lower level than the hormone refractory cell models. Cellular fractionation and immunocytochemistry revealed nuclear localization of AhR in the established hormone refractory cell lines while LNCaP cells are devoid of nuclear AhR protein. qRT-PCR analysis used to assess basal CYP1B1 levels and a xenobiotic responsive element binding assay confirmed ligand independent transcriptional activity of AhR in DU145, PC3 and PC3M cells. Basal CYP1B1 levels were decreased by treatment with specific AhR inhibitor, CH223191. An *in vitro* growth assay revealed that CH223191 inhibited growth of DU145, PC3 and PC3M cells in an androgen depleted environment. Immunohistochemical staining of prostate cancer tissues revealed increased nuclear localization of AhR in grade 2 and grade 3 cancers compared to the well differentiated grade 1 cancers.

**Conclusions:**

Together, these results show that AhR is constitutively active in advanced prostate cancer cell lines that model hormone refractory prostate cancer. Chemical ablation of AhR signaling can reduce the growth of advanced prostate cancer cells, an effect not achieved with androgen receptor inhibitors or growth in androgen depleted media.

## Introduction

In the United States, prostate cancer (PCa) is the most commonly diagnosed cancer in males and the second leading cause of cancer-related death for men [1]. The American Cancer Society estimates that there will be approximately 238,590 men diagnosed with PCa and that 29,720 will die from PCa related causes in 2013 [1]. According to national survival statistics, the five year survival rate for men diagnosed with local or regional prostate cancer is 100%. However, men diagnosed with a distant metastasis have a five year survival rate of just 29% [2].

Since PCa is androgen dependent, the primary treatment involves androgen deprivation therapy (ADT) for metastatic disease [3]. Most prostate cancers initially respond to ADT as measured by a reduction in serum prostate specific antigen (PSA). However, within 2 years most patients stop responding to treatment and develop hormone refractory prostate cancer (HRPC) [4], [5]. There is no cure for hormone refractory prostate cancer (HRPC), which although ADT resistant is still androgen receptor dependent [6]. Numerous mechanisms have been implicated in sustained androgen receptor signaling in HRPC. These include increases in androgen receptor expression, increased steroidogenesis within the tumor cells, point mutations that alter androgen receptor activity, changes in the balance of co-activator/co-repressor proteins, and changes in cell signaling pathways that crosstalk with androgen receptor [5], [7]. Recent findings suggest that the aryl hydrocarbon receptor may participate in crosstalk with AR and support AR growth under androgen deprived conditions. Additionally, studies have shown that AhR has an impact on androgen receptor transcriptional activity. AhR and the AhR-nuclear translocator (ARNT) interact with the androgen receptor [8]. However, only AhR was able to enhance androgen receptor transcriptional activity in the absence of an exogenous ligand [9].

Currently, AhR is the only known ligand-activated member of the basic-helix-loop-helix (bHLH) family of transcription factors. It is activated by the binding of a wide range of environmental toxins including polyaromatic and polycyclic hydrocarbons (PAH) [10]. While in the cytosol, AhR is found in a complex that consist of two molecules of HSP90, co-chaperone p23, immunophilin-like AhR interacting protein (AIP) and tyrosine kinase c-src [11], [12], [13], [14]. This protein complex is designed to maintain the inactive conformation and prevent nuclear translocation.

Upon binding by ligands, activated AhR translocates to the nucleus and heterodimerizes with the AhR nuclear translocator protein (ARNT) [10], [15]. The nuclear AhR complex interacts with xenobiotic response elements (XRE) in the gene promoters of phase I and phase II drug metabolizing enzymes to enhance transcription [16], [17], [18]. Following the induction of AhR responsive genes, AhR signaling is immediately terminated by degradation or by binding by an inhibitor protein [19], [20], [21].

AhR ligand activation has been reported to antagonize androgen receptor signaling. Potent AhR agonist, 2,3,7,8-tetrachloro-dibenzo-*p*-dioxin (TCDD), inhibited testosterone-dependent transcriptional activity and testosterone-regulated prostate specific antigen (PSA) expression in a dose dependent manner [22]. TCDD also inhibits androgen dependent proliferation of prostate cancer cells [23]. Co-activation of AhR and androgen receptor with TCDD and Dihydrotestosterone (DHT) decreased AR protein levels [24]. This observation is contributed to the ability of AhR to promote the proteolysis of AR through assembling an ubiquitin ligase complex in which AhR acts as a substrate-recognition subunit to recruit AR and may explain the antiandrogenic actions of a number of AhR ligands [25].

Despite the studies confirming AhR ligand regulation of AR signaling, AhR may possess intrinsic functions that regulate growth of prostate cancers independent of AR status that has not been fully studied. Structurally, AhR contains both a nuclear localization signal and a nuclear export signal that are required for nuclear-cytoplasmic shuttling of AhR [26]. Several reports reveal constitutive AhR signaling within various cancer types. In the absence of exogenous ligands, AhR overexpression up-regulated the expression of target gene CYP1B1 in the early stage of lung adenocarcinoma [27]. CYP1B1 is also expressed in non-small cell lung cancer cells in the absence of an exogenous ligand. CYP1B1 expression is accompanied by increased AhR expression and constitutive activity of the receptor [28], [29]. Depletion of AhR protein resulted in the subsequent decrease of CYP1B1 expression, confirming that the basal CYP1B1 expression is regulated by constitutive AhR signaling. Pre-malignant and malignant mammary tissues are reported to constitutively express CYP1B1 mRNA. In these human and rodent mammary tumors, AhR was also over-expressed and constitutively active [30].

Additionally, mouse hepatoma cells not exposed to exogenous AhR ligands was shown to contain transcriptionally active AhR. Also, a significant level of constitutive AhR activity was reported in cells isolated from head and neck squamous cell carcinoma (HNSCC) patients (DiNatale2012). Also, transient overexpression of AhR into an AhR null cell line also induced ligand independent transcriptional activity [29], [31].

Prostate tissue analyzed by immunohistochemistry revealed that benign hyperplasia (BPH) epithelial cells possess significantly decreased AhR expression when compared to normal tissue. However, AhR expression was frequently increased in more dedifferentiated tumor areas [32]. A separate study also detected significantly higher AhR expression and activation in tumor cells compared to benign glandular epithelium [33].

The LNCaP cell line, derived from a lymph node metastasis, is a widely used human prostate cancer cell line used to demonstrate androgen sensitivity. LNCaP cells express a mutated androgen receptor and prostate specific androgen [34]. LNCaP cells are not tumorigenic in nude mice [35], [36]. In contrast, androgen insensitive prostate cancer cell lines, DU145 and PC3 are highly tumorigenic in nude mice. Although they do not express the androgen receptor, they are responsive to androgens but do not have repressed growth under androgen deprived growth conditions [37], [38]. These cell lines are commonly used as *in vitro* models for studies involving hormone refractory prostate cancer. The PC3M prostate cancer cell line was isolated from nude mice following intraspenic injection of PC3 cells and is highly metastatic [39]. Although several studies have shown the effects of AhR ligand activation in prostate cancer cell lines, no study has investigated the role of constitutive AhR signaling on prostate cancer cellular growth. We have previously reported that AhR is required to maintain hormone independent signaling and growth by the androgen receptor in C4-2 prostate cancer cells. This evidence shows a direct role for AhR in androgen receptor dependent growth of prostate cancer cells [29]. In this present study we show that AhR is constitutively active in advanced prostate cancer cells and that ablation of constitutive AhR signaling to inhibit androgen independent growth is not dependent on androgen receptor status.

## Materials and Methods

### Chemical and Reagents

AhR agonist, 2,3,7,8-tetrachloro-dibenzo-*p*-dioxin (TCDD) was purchased from AccuStandard (New Haven, Connecticut). AhR antagonist, (CH223191) was purchased from Sigma Aldrich. Androgen receptor antagonist, casodex (CDX) was purchased from Sigma Aldrich.

### Cell Culture

Adherent monolayer cultures of human prostate cancer cell lines LNCaP, DU145, PC3 and PC3M were maintained in RPMI 1640 medium supplemented with 10% FBS and 100 mmol/L each of penicillin and streptomycin. Cells were grown at 37°C with 5% CO2 in humidified atmosphere, and media was replaced every third day. Cells were split (1∶3), when they reached near confluence. Their response to androgens for growth and androgen receptor activity was monitored intermittently during the study.

### RNA Extraction and Quantitative qRT-PCR Analysis

Total RNA was isolated from cell monolayers grown in 100 mm tissue culture dishes using RNeasy Mini Kit (Qiagen). 2 µg of the total RNA was reverse-transcribed using the Superscript II kit (Invitrogen), according to the manufacturer’s recommendations. The cDNA served as a template in a 25 µl reaction mixture and was processed using the following protocol: an initial denaturation at 95°C for 3 min, followed by 39 amplification cycles (95°C for 10 s and 55–65°C for 30 s), 95°C for 10 s, 65°C for 5 s and 95°C for 50 s. The 25 µl qPCR reaction mixture was mixed with GoTaq qPCR Master Mix (Promega). Melt curve analyses were performed after each run to ensure a single product. Relative gene expression was determined using the ΔΔCq calculation method. The primer sequences used were: L-19: Forward (5′-3′) TCCCAGGTTCAAGCGATTCTCCTT & Reverse (5′-30′ TTGAGACCAGCCTGACCAACATGA. CYP1B1: Forward (5′-3′) TGCCTGTCACTATTCCTCATGCCA & Reverse (5′-3′) TCTGCTGGTCAGGTCCTTGTTGAT. The specificity of these primer sets were validated by performing experiments using specific shRNAs that target AhR in Tran et al [29].

### Protein Isolation and Western Blot Analysis

Protein samples were isolated using the Thermo Scientific NE-PER Extraction kit for cellular fractions or commercially available cell lysis buffer (Cell Signaling) for total protein. Protein samples were resolved by SDS-PAGE and transferred to a PVDF membrane. Immunoblotting was carried out with 1 µg/ml mouse AhR monoclonal antibody at 1∶1000 dilution in 5% milk. Blots were washed three times (15 min each) with TBST. The blots were then incubated in 1∶2500 dilution of secondary antibody and washed three times (15 min each) with TBST, three times (10 min each) with TBS and once with ddH20 (10 min). Bands were visualized with the enhanced chemiluminescence (ECL) kit as specified by the manufacturer. Multiple exposures of each set of samples were produced. The relative concentration of target protein was determined by computer analysis and normalized to an internal standard (topoisomerase, β-tubulin, β-actin).

### Immunocytochemical Staining and Fluorescence Microscopy

Cells grown on glass cover slips in 6-well plates were washed in cold PBS and fixed by incubation in a 1∶1 methanol: acetone solution at 4°C for 30 minutes and then air dried. Cells were rinsed and hydrated with Tris-buffered saline containing 0.05% Tween 20 (TBST) and transferred to a clean 6-well plate. The cells were incubated at room temperature for 1 hour in 5% milk solution in TBST to block nonspecific binding, followed by incubation at room temperature for 1 hour with affinity-purified rabbit anti-AhR polyclonal antibody at 1 µg/ml at 1∶1000 dilution in 4% milk solution in TBST. Cells were then washed three times (15 min each) with TBST. Cells were incubated with a 1∶200 dilution of fluorescein isothiocyanate (FITC)-conjugated anti-rabbit antibodies (Jackson Immunoresearch laboratories, West Grove, PA) in 4% milk at room temperature for 1 hour. The cells were then washed three times (15 min each) with TBST, three times (10 min each) with TBS and once with ddH20 (10 min). Cells were then mounted on slides using UltraCruz hard set mounting medium containing 4′6′-diamidino-2-phenylindole (DAPI).

### XRE Binding

4×10^4^ cells were plated in a 96 well plate. Prostate cancer cells were transfected with XRE reporter, as well as with positive and negative control reporter plasmids using attractene. After 18 hours of transfection, media was changed to standard assay media (DMEM +0.5% FBS +0.1 mM NEAA). Cells were grown for an additional 24 hours under normal cell conditions. A dual luciferase assay was performed after 42 hours of transfection, and promoter activity values are expressed as arbitrary florescence units (AFU). Experiments were performed in triplicate and the standard error is indicated.

### Proliferation Studies

Growth of cells were assayed using the Promega CellTiter 96 Cell Proliferation Assay. Cells were resuspended to a final concentration of 1.0×10^5^/mL in RPMI. 50 µl of the cell suspension (5,000 cells) was added to each well of the 96-well plate containing 50 µl of media with corresponding treatment resulting in a total volume of 100 µl. The microplates were incubated at 37°C for 24–72 hours in a humidified, 5% CO_2_ atmosphere. Per manufacturers instructions, following incubation, 20 µl of MTS solution was added to each well and incubated for 4 hours. 100 µl of stop solution was added to each well and incubated for 1 hour. Absorbances were read at 570 nm using the Synergy H1m multimode microplate reader.

### Immunohistochemical Staining

Tissue slides were deparaffinized in xylene and rehydrated in graded down-series of ethanol (70, 90 and 100%) and finally ddH20. Antigens were retrieved using Biocare buffer prior to incubation in 0.3% H_2_O_2_ for 10 minutes at room temperature. Slides were washed three times (5 min each) in PBS. Slides were blocked by incubation in normal goat serum blocking solution for 1hour at room temperature. The slides were incubated with 1 µg/ml rabbit anti-AhR polyclonal antibody (1∶100 dilution) overnight at 4°C. Following incubation with primary antibody, slides were washed three times (5 min each) with PBS prior to a 1 hour incubation with goat, anti-rabbit secondary antibody (1∶400) dilution at room temperature. The slides were washed three times (5 min each) in PBS and incubated 10 minutes with diaminobenzedine per manufactures instructions. Again, slides were washed three times (5 min each) with PBS, rinsed with ddH_2_O and dehydrated in graded up-series of ethanol before being cleared in xylene and mounted using xylene based mounting media. Images of each tissue sample as well as corresponding hematoxylin and eosin stains were captured at 400x magnification for subsequent scoring. Anti-AhR reactivity was scored on a scale of 1–3 (1 = low reactivity and 3 = high reactivity) for the cytoplasm and nucleus of each tissue sample by two independent investigators.

### Statistical Analysis

Each experiment was carried out at least 3 times and all the values are expressed as mean +SEM. The differences between the groups were compared by t-test or ANOVA using InStat software (GraphPad Software Inc., San Diego, CA). A value of P<0.05 was considered statistically significant.

## Results

### I. AhR is Overexpressed in Advanced Prostate Cancer Cell Lines

DU145, PC3 and PC3M prostate cancer cell lines were used as hormone refractory prostate cancer cell models. These 3 cell lines have been shown to maintain growth rates in an androgen depleted environment [37], [38], [39]. LNCaP is an androgen sensitive prostate cancer cell model whose growth rate is reduced under androgen depleted conditions [34]. The expression of AhR mRNA in the cell lines was quantified by qRT-PCR. AhR protein expression of each line was examined by western blot. Advance prostate cancer cell lines have an increase in the expression of AhR mRNA and protein compared to the androgen sensitive, LNCaP, cell line. LNCaP cells express both AhR mRNA and protein. However, DU145 and PC3 cell have a 2.5 and 5 fold increase in AhR mRNA respectively (Fig. 1B). This correlates with the 2 fold increase in AhR protein in DU145 and the more than 2.5 fold increase in PC3 cells (Fig. 1A). PC3M cells have the largest increase in AhR expression when compared to LNCaP cells. There was a 10 fold increase in PC3M mRNA and 3-fold increase in AhR protein (Fig. 1).

**Figure 1:** AhR mRNA and protein expression in prostate cancer cell lines. **A.** Total cellular proteins were isolated from LNCaP, DU145, PC3 and PC3M prostate cancer cell lines. Proteins were separated by SDS polyacrylamine gel electrophoresis and blotted using an anti-AhR antibody. Anti-β-actin was used as a loading control. Image J was used to obtain desitometric measures from 3 independent membranes. Each bar represents mean±SEM (n = 3) and were analyzed by student t-test. Statistically significant differences (*p<0.05) compared to LNCaP control. **B.** Total RNAs were isolated and quantitative RT-PCR was performed to determine the mRNA expression of AhR in the prostate cancer cell lines. mRNA levels were normalized using L-19 which serves as an internal control. Each bar represents mean±SEM (n = 3) and were analyzed by student t-test. (*) denotes statistically significant differences between groups.

### II. Ligand Independent Nuclear Localization of AhR

To determine localization of AhR protein, we isolated cellular fractions and performed immunoblotting for AhR in the nuclear and cytoplasmic fractions. Western blot analysis of cellular fractions revealed that the increase AhR expression in the advanced prostate cancer cell lines is accompanied by nuclear accumulation of AhR without stimulation by an exogenous ligand. Although AhR protein was detected in the cytoplasmic fractions of LNCaP cells, no AhR was detected in LNCaP nuclear fractions. In contrast, the advanced prostate cancer cells lines showed high expression of the AhR protein in the nuclear fractions (Fig. 2A). Immunocytochemistry confirmed the presence of AhR in the nucleus of DU145, PC3 and PC3M cells. The absence of any staining overlay in the merged image of the DAPI stained nuclei and FITC-stained AhR further demonstrated that LNCaP cells do not possess nuclear AhR (Fig. 2B).

**Figure 2:** Subcellular localization of AhR in prostate cancer cells. **A.** Nuclear and cytoplasmic fractionation: Cell lines were grown on 100 mm dishes until ∼75% confluent, washed with cold PBS and cellular fractions were isolated by per manufactures instructions using a NE-PER Extraction kit. The nuclear and cytoplasmic fractions were analyzed by western blotting for AhR protein expression. The relative level of cytoplasmic AhR was normalized with β-tubulin expression and the relative level of nuclear AhR was normalized with topoisomerase expression. Bars represent mean±SEM of the corrected values from three independent experiments and (*) denotes constitutive nuclear levels of AhR that are significantly different between cell lines. **B.** Subcellular localization of AhR in prostate cancer cell lines by immunocytochemical staining: Cells were grown on coverslips and fixed with methanol:acetone. AhR was visualized by staining with rabbit anti-AhR polyclonal antibodies followed by FITC-conjugated goat anti-rabbit antibody. The nuclei were counter-stained with DAPI fluorescence dye. Images from FITC and DAPI-fluorescence channels were merged. Images were captured on an Olympus wide fluorescence microscope (400x magnification).

### III. Constitutive AhR Transcriptional Activity

The Cignal XRE reporter was used to measure the basal activity of the AhR signaling pathway in advanced prostate cancer cell lines. The assay used to test AhR promoter activity revealed that the advance prostate cancer cells DU145, PC3 and PC3M, all possess a high level of AhR binding to XRE in the absence of an exogenous ligand. The androgen sensitive LNCaP cell line demonstrated minimal XRE binding. PC3 cells demonstrated the highest promoter activity with an 10-fold increase in XRE binding compared to the LNCaP cell lines. DU145 and PC3M cells demonstrated an 2.5 and 8-fold increase in promoter activity compared to the LNCaP cell line, respectively (Fig. 3A).

**Figure 3:** Constitutive AhR transcriptional activity in advanced prostate cancer cell lines. **A.** Each prostate cancer cell line was transfected with an XRE reporter plasmid, as well as with positive and negative control reporter plasmids using attractene. Following transfection, a dual luciferase assay was performed. Promoter activity values are expressed as arbitrary florescence units (AFU). Each bar represents mean±SEM (n = 3) and were analyzed by student t-test. (*) denotes statistically significant differences (*P<0.05). **B.** qRT-PCR analysis of CYP1B1 mRNA expression in prostate cancer cells. Cells were treated with 50 µM of AhR inhibitor (CH223191) or vehicle control (DMSO) for 24 h and total RNAs were isolated and quantitative RT-PCR was performed to determine the mRNA expression of CYP1B1 in each prostate cancer cell lines. mRNA levels were normalized using L-19 which serves as an internal control. Each bar represents mean±SEM (n = 3) and were analyzed by student t-test. (*) denotes statistically significant differences (*P<0.05) compared to LNCaP prostate cancer cell line.

The above results suggest a transcriptionally active AhR in advanced prostate cancer cell lines. Several reports have confirmed elevated AhR and CYP1B1 but not CYP1A1 in tumorigenic models [30], [40]. These studies suggest the existence of differences in regulation of these two genes. CYP1A1 and CYP1B1 expressions are both AhR mediated but differences in promoter structure may result in differential expression. The reports indicate that CYP1A1 is control by ligand activation of AhR and CYP1B1 is regulated by constitutive AhR signaling [41], [42], Therefore, to confirm transcriptional activity of the AhR signaling pathway, AhR responsive gene, CYP1B1 was measured by qRT-PCR in the androgen sensitive LNCaP cell line as well as the advanced prostate cancer cell lines, DU145, PC3and PC3M. LNCaP cells expressed minimal levels of CYP1B1 transcript. DU145 and PC3 cells demonstrated a 12 and 25-fold increase in CYP1B1 when compared to the LNCaP cells. PC3M cells demonstrated the largest fold increase in CYP1B1 with a almost 30 fold increase compared to LNCaP cells. Inhibition of AhR signaling by direct inhibitor, CH223191, resulted in a substantial decrease in CYP1B1 levels in the advanced prostate cancer cell lines. Due to the low basal expression of CYP1B1 in LNCaP cells, CH223191 had no significant effect on CYP1B1 mRNA expression (Fig. 3B).

### IV. Ablation of Constitutive AhR Signaling Inhibits Androgen Independent Growth

The above data demonstrates the ability of AhR antagonist, CH223191, to inhibit constitutive AhR signaling. To determine the effect of constitutive AhR signaling on the growth rate of advanced prostate cancer cells, each cell line was grown in the absence and presence of the specific AhR inhibitor, CH223191. LNCaP, DU145, PC3 and PC3M prostate cancer cells were grown in the presence of AhR inhibitor CH223191191 in concentrations ranging from 1 µM to 50 µM (Fig. 4A). Ablation of AhR signaling was sufficient to reduce the growth rate of all cell lines including the androgen sensitive LNCaP cells. To confirm the effects of CH223191191 were AhR dependent, DU145 cells were transfected with a control vector (SCR) and a vector carrying specific shRNA to target AhR protein (-AhR). The resulting cells that express AhR (SCR) and are devoid of AhR protein (-AhR) were treated with 50 µM CH223191191 (Fig. 4B). The DU145 (SCR) cells respond to CH223191191 treatment with a significant decline in growth rate while the DU145 (-AhR) cells exhibited no growth response to the AhR antagonist (Fig. 4B). Androgen receptor inhibition by casodex was only effective in LNCaP cells. Treatment of advanced prostate cancer cell lines (DU145, PC3 and PC3M) with CDX had no effect on growth rate. LNCaP cells exhibited a 40% decrease in growth rate in the presence of CDX. CH223191 treatment resulted in the largest growth inhibition in DU145 cells. DU145 cells also demonstrated the highest growth rate of all cell lines under control conditions. Also, co-treatment with CH223191 and CDX resulted in an additional decrease in growth rate compared to CH223191 alone in all cell lines (Fig. 4C). Growth inhibition of the prostate cancer cell lines by CH223191191 remained for up to 72 hours (Fig. 4D).

**Figure 4:** Inhibition of AhR signaling decreases growth of prostate cancer cells. **A.** Cells were grown in a 96 well plate at 5.0×10^3^ cells per well. The cells were treated with DMSO or 1 µM, 5 µM, 10 µM, 25 µM or 50 µM of CH223191. Cell growth was measured using Promega CellTiter 96 Cell Proliferation Assay per manufactures instructions. **B.** Confirmation of AhR protein expression in DU145 cells with scrambled vector control (SCR) and shRNA lentivirus against AhR (-AhR) by western blotting. 20 µg of protein isolated from was analyzed by western blotting. β-action is used as a loading control. Proliferation of DU145(SCR) and DU145(-AhR) cells were analyzed using the CellTiter 96 Cell Proliferation Assay in the presence and absence of 50 µM of CH223191. **C.** The cells were grown in charcoaled stripped media and treated with DMSO (CON), 20 µM casodex (CDX), 50 µM CH223191 or a combination of CDX and CH223191 for 72 hours. Cell growth was measured using Promega CellTiter 96 Cell Proliferation Assay per manufactures instructions. Each bar represents mean±SEM (n = 3), *p<.05. **D.** Cells were serum starved for 24hrs and grown in charcoal stripped (CSS) media. Cells where then treated with DMSO (Con) or 50 µM CH223191 for an additional 24, 48 or 72 hours. At each endpoint, cells were analyzed for DNA content using the cell proliferation assay as described in the materials and methods. Each data point represents mean±SEM (n = 3). (*) denotes a significant difference compared to respective DMSO control.

### V. AhR Nuclear Accumulation in Prostate Cancer Tissue

The expression and localization of AhR was assessed in prostate cancer tissue by immunohistochemical staining. In line with the objective of this study to show that AhR is constitutively active in advanced prostate cancer, we assessed AhR expression in prostate cancer tissues ranging from Grade 1 to Grade 3. Grade 1 tissues are well differentiated and the cells appear normal. Grade 2 tissues are moderately-differentiated and the cells appear slightly different than normal. Grade 3 tissues are poorly differentiated and the cells appear abnormal and tend to grow and spread more aggressively. 100% of the tissues stained positive for cytoplasmic AhR. However, only 14% of grade 1 tissues were positive for nuclear AhR compared to 50% of grade 2 and grade 3 cancer tissues (fig. 5A and table 1). The presence of nuclear AhR in grade 2 and grade 3 tissues along with the in vitro data from the prostate cancer cell lines suggest a transcriptionally active AhR in these higher grade tumors. Additionally, all grade 1 tumors positive for nuclear AhR were all classified as Stage IV tumors. Analysis of total AhR expression revealed that Grade 2 and 3 tumors possess significantly more total AhR compared to grade 1 tissue (fig. 5B). In addition, ∼80% of tissues with Gleason score 7 or greater have increased anti-AhR reactivity compared to only 47% of tissues with Gleason score 2–6 (Table 2).

**Figure 5:** AhR expression in prostate cancer tissues. **A.** Representative Grade 1, Grade 2 and Grade 3 prostate cancer tissues: Upper panel stained with anti-AhR polyclonal antibody; lower panel stained with hematoxylin and eosin. The arrows depict positive anti-AhR reactivity in the nucleus of grade 2 and grade 3 tumors. **B.** Total anti-AhR reactivity was scored in grade 1, grade 2 and grade 3 prostate cancer tissues based upon intensity level in both cytoplasm and nucleus (0–1). Total AhR score was determined by combining individual cytoplasmic and nuclear scores.

**Table 1:** Cytoplasmic and nuclear expression of AhR in prostate cancer tissues.

Grade	% Cyto AhR	%Nuc AhR
1	100%	14%
2	100%	50%
3	100%	50%

Immunohistochemistry revealed anti-AhR reactivity in the cytoplasm of all grades of prostate cancer tissues stained and increased reactivity in the nucleus of grade 2 and grade 3 tumors.

**Table 2:** AhR reactivity by Gleason score: Prostate cancer tissues were catorized based upon Gleason score 2–6 (well differentiated), 7 (moderately differentiated) or 8–10 (poorly differentiated).

Gleason Score	AhR Score 0–1	AhR Score 2–3
2–6	53%	47%
7	22%	78%
8–10	20%	80%

The percent anti-AhR activity for each category is listed based upon low (0–1) or high (2–3) total AhR score.

## Discussion

Several studies suggest AhR promotes proliferation in the absence of exogenous ligands, whereas treatment with exogenous ligands inhibits cellular proliferation. A study on the ovulation rate in rats following TCDD exposure revealed that AhR ligand activation induces a G2/M cell cycle block resulting in a decrease in S-phase cells. This study also found that TCDD inhibits levels of Cdk2 and cyclin D2 [43]. The inhibitory effect has been seen with both genotoxic and non-gentoxic ligands for AhR. Microarray analysis of LNCaP prostate cancer cells treated with genotoxic ligand benzo[a]pyrene (BaP) and nongenotoxic ligand 2,3,7,8-tetrachlorodibenzo-p-dioxin (TCDD), revealed a significant overlap in both up-regulated and down-regulated genes. Both AhR ligands suppressed expression of genes associated with cell cycle progression and DNA replication [44]. Mice treated with TCDD following injection of mammary tumor cells experienced a 50% decrease in metastasis to the lung as well as in secondary mammary gland sites compared to non-treated mice. Interestingly, primary tumor growth was not affected by TCDD treatment [45].

AhR ligands have also been shown to inhibit proliferation of PCa cells in the presence of androgens. Co-treatment of LNCaP cells with DHT and TCDD decreased AR protein levels in addition to decreasing growth rate [24]. Diesel exhaust particles, confirmed to be AhR agonist, inhibit DHT induced androgenic effects in PC3 prostate cancer cells. The antiandrogenic effects of the diesel exhaust particles was reversed by treatment with AhR antagonist, a-naphthoflavone [46]. The antiandrogenic effect of AhR ligands chrysene (Chr), benzo[k]fluoranthene (BkF), benzo[a]pyrene (BaP) were studied in LNCaP prostate cancer cells. All three ligands exhibited an antiandrogenic effect by inhibiting DHT induced PSA mRNA and protein levels. alpha-Naphthoflavone (alpha-NF), an AhR antagonist, reversed the antiandrogen action of Chr, BkF and BaP, suggesting a requirement for activated AhR [46]. Chlorinated byphenyls, also known AhR ligands, exhibited antiandrogenic properties by reducing androgen stimulated PSA and cell proliferation of LNCaP cells. These AhR ligands also inhibited the DHT-producing enzyme 5-α-reductase [47].

2,3,7,8-Tetrachlorodibenzo-p-dioxin (TCDD) and related compounds can modulate proliferation by enhancing ligand metabolism, altering hormone synthesis, down regulating receptor levels, and interfering with gene transcription. TCDD has been shown to inhibit both normal and testosterone-stimulated growth; testosterone treatment also dose-dependently inhibited TCDD-induced transcriptional activities [22]. A separate study investigating the mechanism for DHT inhibition of AhR transcriptional activity revealed that the protein levels of AhR and AhR nuclear translocator (ARNT) were not affected by DHT. However, the inhibitory effect of DHT was abolished by knockdown of the androgen receptor protein with siRNA. It was determined that DHT induced heterodimerization between AR and AhR when cells were also treated with an AhR agonist [48]. The data presented here, reveals that AhR can modulate proliferation of prostate cancer cells in the absence of androgen receptor. DU145, PC3 and PC3M cells do not express the androgen receptor and all have constitutive AhR signaling that maintains the growth rate of these cultured cells.

In vitro studies have demonstrated that in human breast cancer cells AhR, cyclin D1 and cyclin dependent kinase 4 (CDK4) interact within the cell cycle and the interaction was disrupted upon TCDD treatment. CDK4 kinase activity assays demonstrated that retinoblastoma (Rb) phosphorylation regulated by the AhR/CDK4/cylinD1 complex was reduced in the presence of TCDD and correlated with a G1 cell cycle arrest [49]. These results indicate that the AhR interacts in a complex with CDK4 and cyclin D1 in the absence of exogenous ligands to facilitate cell cycle progression and explains the opposing role of AhR ligand activation and expression on cell cycle regulation.

Despite the overwhelming evidence of anti-proliferative activities of AhR ligands, accumulating evidence suggest that in advanced stages of prostate cancer AhR is constitutively active and may promote progression [49], [50], [51]. Competition binding assays have confirmed true ligands for AhR. Both the indole metabolite, indoxyl 3-sulfate (I3S) and kynurenic acid, a metabolite of the indoleamine-2,3-dioxygenase pathway have been identified as endogenous AhR ligands [52]. However, their expression and activity needs further investigation and may ultimately provide further insight into the constitutive AhR signaling observed in advanced staged cancers.

Irrespective of the discovery of several endogenous ligands, accumulating evidence shows that modulation of AhR protein expression directly correlates with disease progression. A resulting increase in AhR expression by retroviral expression vectors in mammary epithelial cells correlated with the development of cellular malignant phenotypes. Clones overexpressing AhR exhibited increased proliferation due to enhanced cell cycle progression. In addition, cells overexpressing AhR exhibited enhanced migration as well as the ability to invade matrigel matrix [50]. Conversely, AhR depleted clones of the human breast cancer cell line MDA-MB-231 attenuated tumorigenic properties *in vitro* including proliferation, anchorage independent growth, migration and apoptosis. Subsequent analysis revealed AhR knockdown significantly reduced phosphorylation of AKT, which impacts cell proliferation and survival [53].

Granule neuron precursors (GNPs) which give rise to medulloblastoma express high levels of the AhR. Studies show that either abnormal activation or deletion of the AhR leads to dysregulation of GNP cell cycle activity and maturation. Compared with wild-type medulloblastoma tumor cells, AhR shRNA medulloblastoma tumor cells displayed an impaired G(1)-to-S cell cycle transition, decreased DNA synthesis and reduced proliferation. Supplementation experiments with human AhR restored the proliferative activity [51]. Immunoblot analysis showed that AhR expression is increased in androgen independent (C4-2) prostate cancer cells when compared to androgen sensitive (LNCaP) cells. RT-PCR studies revealed constitutive AhR signaling in C4-2 cells without the ligand induced activation required in LNCaP cells. A reduction of AhR activity by short RNA mediated silencing in C4-2 cells reduced expression of both AhR and androgen responsive genes. The decrease in androgen responsive genes correlates to a decrease in phosphorylated androgen receptor and androgen receptor expression in the nucleus. Furthermore, the forced decrease in AhR expression resulted in a 50% decline in the growth rate of C4-2 cells [29]. Previous studies have determined an androgen dependent role for AhR in prostate cancer growth. This current study reveals AhR’s ability to modulate growth of prostate cancer cells independent of androgen receptor activity. Further studies are needed to determine the effect of increased AhR expression on CDK4 activity in advanced prostate cancer cells. The ability of constitutive AhR signaling to regulate cell cycle progression in advanced prostate cancer cells makes AhR a possible target for treatment of HRPC.
